# Bariatric Surgery in Rats Upregulates FSP27 Expression in Fat Tissue to Affect Fat Hydrolysis and Metabolism

**DOI:** 10.1155/2019/6415732

**Published:** 2019-05-08

**Authors:** Jingyao Hu, Mofei Wang, Yong Zhou, Xiaowei Zhang, Bing He, Lei Liu, Rui Ma, Tianyi Zhang, Keyi Liu, Yong Wang, Jingang Liu

**Affiliations:** ^1^The Fourth Affiliated Hospital of China Medical University, 110032 Shenyang, China; ^2^Shengjing Hospital affiliated to China Medical University, 110004 Shenyang, China

## Abstract

**Purpose:**

To explore the changes in FSP27 expression and fat metabolism in adipose tissue and their relationship after bariatric surgery in rats.

**Method:**

Food intake, body weight, triglyceride content, fat distribution, and fat cell morphology were evaluated in rats grouped into control, sham, sleeve gastrectomy (SG), and Roux-en-Y gastric bypass (RYGB) groups. Immunohistochemistry and western blotting were used to detect protein expression and real-time PCR was used to detect mRNA expression. Mouse 3T3-L1 preadipocytes were used to assess the effects of different energy levels and nutrient factors on FSP27 in adipocytes.

**Result:**

Food intake, body weight, and triglyceride levels were reduced in RYGB and SG rats within 28 days after surgery, with a more pronounced effect in the RYGB group. Weight loss was mainly due to loss of fat mass rather than loss of lean mass, with the most pronounced decrease in trunk fat. FSP27 expression increased in lean rat adipocytes accompanied by increased lipid droplets (LDs). In SG and RYGB rats, the FSP27 protein concentration gradually increased in white adipose tissue (WAT) after operation. Hormone-sensitive lipase (HSL), p-HSL/HSL, Adipose Triglyceride Lipase (ATGL), and Comparative Gene Identification-58 (CGI-58) gradually decreased in SG and RYGB rats, but they were always higher than in control and sham animals. FSP27 was also decreased in 3T3-L1 adipocytes of animals with a high-energy diet.

**Conclusion:**

FSP27 is associated with rat lipid metabolism and its expression varies with energy and nutrient supply. It can inhibit excessive hydrolysis and fat accumulation by regulating HSL and ATGL expression and by mediating LDs formation.

## 1. Introduction

Adipose is the main tissue for storing energy in the body, and it plays an important role in maintaining energy metabolism balance and homeostasis. Fat metabolism disorders can cause diseases such as obesity, fatty liver, and hyperlipidemia. The number of morbidly obese patients rises each year. The World Health Organization (WHO) reported that 39% of adults aged 18 years and over were overweight in 2016, and 13% were obese (https://www.who.int/news-room/fact-sheets/detail/obesity-and-overweight). Through bariatric surgery, obese patients can reduce weight, improve quality of life, and decrease obesity complications [1–3].

Metabolic disorders, especially lipid metabolic disorders, are major factors for obesity. Lipid metabolism intimately involves surface proteins on LDs, which may present drug targets for treating obesity [4, 5]. FSP27 is a LDs-related protein and one of three cell death-inducing DFF45-like effector (CIDE) family proapoptotic proteins. FSP27 is linked to metabolic diseases such as human obesity, diabetes, and fatty liver. FSP27 is abundantly present in white adipose tissue and brown adipose tissue (BAT) [6–9], and it can promote small LDs fusion and block fat hydrolysis [10–12]. FSP27 has antilipolytic activity, and it is essential for fat cells to store triglycerides [6–8, 13–16].

Many studies report that FSP27 affects lipolytic enzymes. FSP27 was confirmed to inhibit enzyme localization on LDs by direct or indirect interaction with HSL and ATGL thereby inhibiting lipolysis and promoting triglyceride storage in fat cells [13, 15–18]. Some have reported that calorie restriction inhibits FSP27 expression in mouse epididymis adipose tissue [19]. Decreased caloric intake may lead to a similar decrease of FSP27 in humans [20] when fat cells adapt to systemic energy deficiency [20, 21]. However, FSP27, HSL, and ATGL were increased in subcutaneous and visceral fat in bariatric surgery patients with reduced dietary intake and weight loss [22, 23]. Whether FSP27 participates in and effectively regulates lipid metabolism in individuals with rapidly decreasing body weight has not been elucidated in detail.

This study investigated FSP27-mediated regulation of lipid synthesis and decomposition and its effect on energy homeostasis in adipose tissue of obese and lean rats. Animal experiments confirmed dynamic expression changes of FSP27 in rat adipose tissue after bariatric surgery and its regulation of downstream protein and fat metabolism. Cell experiments further validated the influence of the nutrient and energy environment on FSP27 protein expression in 3T3-L1 adipocytes. We aimed to investigate the effects of bariatric surgery on FSP27 levels and the relationship between FSP27 and fat metabolism.

## 2. Materials and Methods

### 2.1. Laboratory Animals and Grouping

Male Sprague-Dawley rats, 4-6 weeks old, weighing 220~230g and high-fat diet were purchased from Beijing Huafukang Biotechnology Co., Ltd. Animal experiments were conducted at the Animal Center of Shengjing Hospital affiliated with China Medical University (CMU), and this experiment was approved by the Animal Welfare Ethics Committee of CMU (NO. 2017010). Diet-induced obesity was used to feed rats with 45% high-fat diet (containing 45% fat, 20% protein, and 35% carbohydrate) as described by Woods et al. [24]. Rats were randomly divided into four groups including obesity (control, n=10), obesity sham surgery (Sham, n=10), obese stomach sleeve gastrectomy (SG, n=10), and obese Roux-En-Y gastric bypass surgery (RYGB, n=10).

### 2.2. Obesity Induction and Surgery

Preparation of the SG group: Rats were anesthetized by intraperitoneal injection of 1% sodium pentobarbital (30 mg/kg). A midline abdominal incision of approximately 3 cm was made, followed by transection of connective tissue attachments to the liver and spleen to isolate the stomach. Following the greater curvature of stomach, from the angle of His in the cardia to 1 cm above the pylorus, approximately 70% of the stomach containing the entire fundus was removed and the remaining tubular section was left to connect the esophagus and pylorus. The residual stomach was sutured and returned to the abdominal cavity; then the abdominal wall was closed.

Preparation of RYGB group was as follows. Rats were anesthetized with pentobarbital sodium, an abdominal incision of approximately 3 cm was made, the small curved side of the stomach at 2-3 mm below the gastroesophageal junction was cut off, and the distal and proximal stomach were sutured. Approximately 20% of the stomach was retained. A 5-8 mm incision was then made in the stomach wall above the gastric sac suture and the jejunum was cut 15 cm from the Treitz distal end and then the distal jejunum was connected to the gastric sac by end-to-end anastomosis. End-to-side anastomosis connected the proximal jejunum to the jejunum 10 cm distal to the gastrojejunal anastomosis. Rats in the sham group had a 1.5-2 cm incision on the greater curvature of the stomach, which was then sutured in situ. Carolyn (5 mg/kg i.p.) was given intraoperatively for analgesia and then administered daily until 1 week after surgery. After the operation, all rats were fasted for 24 hours and then freely given a high-fat diet and water.

### 2.3. Dual-Energy X-Ray Absorptiometry (DEXA)

Rats in each group were anesthetized with 1% pentobarbital sodium (30 mg/kg) intraperitoneally on the 28th day after surgery. The rats were placed on the ventral side and then scanned by DEXA (CUSTOMER: GE Healthcare PRAT#LU0219_01 S/ N: 41666). Results were analyzed using Hologic Apex Software (version3.2, USA).

### 2.4. Measurement of Weight and Food Intake

Rats were weighed on the day of surgery and the 7th, 14th, 21st, and 28th days after surgery. Total food intake and remaining food were recorded weekly to calculate average daily intake. Food and water were readily available throughout the experiment.

### 2.5. Detection of Triglycerides

On the 28th day after surgery, blood was collected from the small saphenous vein of the hind limbs; then epididymal fat, perirenal fat, and interscapular fat tissue were collected, part was fixed in 10% paraformaldehyde, and part was stored immediately at −80°C. Plasma and adipose tissue triglycerides were detected using a triglyceride test kit (GPO-PAP Enzyme Method, Nanjing Jiancheng Bioengineering Institute, Nanjing, China).

### 2.6. Immunohistochemistry

Epididymal fat, perirenal fat and interscapular fat tissue fixed in 10% paraformaldehyde were dehydrated by alcohol gradient, embedded in wax, sliced, baked, dewaxed, microwaved to retrieve antigen, blocked with skim milk for 2 h, and then incubated with Anti-CIDE-C antibody (1:200; Abcam, Cambridge, MA, #198204) overnight at 37°. After washing, biotinylated goat anti-rabbit IgG were added; then streptomycin avidin-peroxide Enzyme (MXB, Fuzhou, China) was added. Slides were exposed to light for 5 min with DBA at room temperature, washed 3 times with PBS for 5 min, counterstained by hematoxylin for 3 min, dehydrated, and then sealed with neutral gum.

### 2.7. Real-Time RT-PCR

The expression of FSP27 and uncoupling protein (UCP1) was detected by real-time PCR. *β* actin was used as the reference gene [25]. Primers were synthesized by Shanghai Shenggong Bioengineering Co., Ltd., and primer sequences are shown in Table 1. We took an appropriate amount of adipose tissue, extracted total RNA with an RNAiso Plus Kit (Takara Biotechnology (Dalian) Co., Ltd.), ran a reverse transcription cDNA kit (Thermo, K1622), and prepared for reaction using a qRT-PCR kit (Qiagen, 204057). The PCR program ran as follows: incubation at 95°C for 30s, then incubation at 95°C for 5s, 60°C for 30 seconds, and repeated 40 cycles. Results were calculated using the 2^∧^(-Delta Delta CT) method.

### 2.8. Western Blotting Assay

To study differential protein expression upon weight loss in rats, a second round of rat obesity and weight loss experiments was run with the same groups (control, sham, SG, and RYGB), with tissue harvested 14 days after surgery. White fat (epidemic fat, perirenal fat) and brown adipose tissue were collected and added to precooled tissue protein lysate to prepare for homogenate via tissue homogenizer. Protein content was detected using a BCA protein detection kit; then proteins were separated by SDS-polyacrylamide gel electrophoresis and transferred to PVDF membranes (1703930, BIO-RAD, USA). After blocking with skim milk for 2 h, HSL, P-HSL/HSL, CGI-58, ATGL, DGAT1, or DGAT2 primary antibody was added. The membrane was developed by ECL luminescence (35050, Pierce, USA). All samples were repeated three times for statistical analysis. Gels were imaged and values were calculated using Image J software (NIH, Bethesda, MD, USA).

### 2.9. Cell Cultivation and Differentiation

Mouse 3T3-L1 preadipocytes purchased from the Institute of Biochemistry and Cell Biology, Chinese Academy of Sciences, were cultivated in DMEM (high glucose formulation; Gibco-BRL) supplemented with 10% heat inactivated FBS in a humidified atmosphere of 5% CO_2_ at 37°C with medium changed every 2-3 days.

To induce 3T3‐L1 differentiation, 3T3‐L1 preadipocytes were grown to confluence. Two days after reaching confluence, cells were induced to differentiate (designated as day 0) by adding a standard differentiation cocktail (DMI) consisting of 0.5 mM 1‐methyl‐3‐isobutyl‐xanthin (IBMX) (Sigma–Aldrich), 1 *μ*M dexamethasone (Dex) (Sigma–Aldrich), and 1 *μ*g/ml insulin (Sigma–Aldrich) to the culture medium. After 2 days, the medium was replaced with DMEM containing 10% FBS and 1 *μ*g/ml insulin, and the cells were incubated for another 2 days. Thereafter, the cells were cultured in DMEM with 10% FBS, with media changed one or two days before full differentiation.

Cell differentiation was determined by Oil Red O staining: cells were fixed in 10% formaldehyde in PBS for 20 min, rinsed with 70% alcohol, stained with Oil Red O for 10 min, rinsed with deionized water, and then observed under a microscope.

FSP27 is highly expressed in mature adipocytes [26], so mature 3T3-L1 adipocytes were induced in high-fat low-sugar medium (containing 0.5mmol/l palmitic acid, 1 g/l glucose, and 10% FBS), high-sugar medium (containing 4.5g/l glucose, 10% FBS), high-nutrient low-sugar medium (containing 1 g/l glucose, 30% FBS), and low-sugar medium (control group, containing 1 g/l glucose, 10% FBS). After 48 hours in culture, western blotting and immunofluorescence were performed.

### 2.10. Immunofluorescence

After dewaxing, tissue sections were washed 3 times in PBS, permeabilized in 0.1% Triton for 10 minutes, subjected to antigen retrieval in citric acid solution, blocked with 5% BSA for 1 hour, and incubated with primary antibody (FSP27/CIDE-C, 1:100, Abcam, Cambridge, MA, #198204) overnight at 4°C. The next day, a secondary antibody (FITC-conjugated goat anti-rabbit IgG, ZSGB-BIO, ZF-0311, 1/150) was added. Cell nuclei were stained with DAPI. Sections were imaged using a fluorescence microscope (Olympus Corporation, Japan).

### 2.11. Statistical Analysis

All data were obtained from experiments repeated at least 3 times, and data analysis was performed using SPSS 20.0 (SPSS Inc., Chicago, IL, USA). Results are expressed as mean ± SD. A two-tailed Student's t-test based on ANOVA was used for 2-group comparisons. P < 0.05 was considered statistically significant.

## 3. Results

### 3.1. Bariatric Surgery Reduces Food Intake, Body Weight, and Triglyceride Levels in Rats

Compared with the obese control group, rat food intake decreased after bariatric surgery. This was more pronounced in the RYGB and SG groups even at 4 weeks after surgery (Figure 1(a)). Rat weight in the SG and RYGB groups decreased by 15.4% and 24.4%, respectively (Figure 1(b)), indicating that the rats reduce food intake and lose weight within 28 days after surgery (Figures 1(a) and 1(b), p<0.05), especially following RYGB. SG and RYGB reduced triglyceride levels in rat plasma and adipose tissue (Figures 1(c) and 1(d)). Bariatric surgery can lead to weight loss by promoting triglyceride breakdown in fat cells.

### 3.2. Trunk Fat Mass of Rats Was Reduced after Operation

Rat body composition was measured by DEXA on postoperative day 28 (Figure 1(a)). The fat mass of SG and RYGB rats was noticeably lower than that of sham and obese controls, while lean mass was not significantly different between the groups (Figures 2(b) and 2(c)). Compared with the control group, the sham, SG, and RYGB groups had lower body fat/body weight percentages, with SG and RYGB notably lower than the sham group (p<0.05). There was no statistical difference between SG and RYGB (Figure 2(d), P > 0.05). The trunk/body fat ratio (%, (Upper limb + thigh) / trunk fat) shows that SG and RYGB rats had a lower proportion of trunk fat (P < 0.05, Figures 2(e) and 2(f)). The above results indicate that rat weight loss after bariatric surgery was mainly due to decreased fat mass, not lean mass, with the most pronounced decrease seen in trunk fat. This indicates that adipose tissue is redistributed during weight loss in rats.

### 3.3. FSP27 Expression and the Number of LDs Number Increase in the Fat of Lean Rats

DEXA detection showed that lean rats pronouncedly reduce trunk fat. We speculated that trunk adipose tissue has a higher metabolic activity during weight loss. To test this, we harvested white fat (epidemic fat, perirenal fat) and brown fat between the shoulders four weeks after the operation according to the body region division in DEXA. Immunohistochemistry showed deeper brown pigmentation in the epididymis, perirenal, and interscapular adipose tissue of SG and RYGB rats (Figure 3(a)). However, FSP27 expression in control and sham rats was nearly unchanged. We observed a large single compartment LDs and the interscapular fat showed the classic multichamber LDs structure of brown fat cells. At 4 weeks after surgery, the trunk fat cells lacked larger LDs due to the higher FSP27 content. On the contrary, lean rat adipocytes showed multicompartment LDs and smaller cell diameters, suggesting that fat cells have strong decomposition activity and heat production function. Real-time RT-PCR showed gene levels of the LDs-related protein FSP27 and brown fat marker protein UCP1 (Figure 3(b)). The increased expression of UCP1 in white fat in SG and RYGB rats confirmed the existence of “browning”. FSP27 expression also increased, which was reported to promote LDs fusion and to decrease the LDs number [10–12], but the LDs in fat cells still increased.

### 3.4. FSP27 May Regulate Fat Hydrolysis in Rats to Prevent Postoperative Weight Loss

Immunohistochemistry and real-time RT-PCR results suggested that FSP27 was upregulated in lean rat fat, which is contrary to previous belief. Western blotting showed downregulated FSP27, DGAT1, and DGAT2 at 2 weeks after surgery in SG and RYGB rats compared with sham and control. HSL, P-HSL/HSL, CGI-58, and ATGL were upregulated in epididymal and perirenal fat. At 4 weeks after surgery, FSP27 protein expression in the adipose tissue of SG and RYGB rats was pronouncedly higher than that of the sham and control groups. HSL, p-HSL/HSL, CGI-58, and ATGL were still higher than sham and control groups in the same period. There was no statistical difference in DGAT1 and DGAT2 across the four groups (Figures 4(a) and 4(b) p>0.05). Perirenal adipose tissue showed similar results to epididymal fat (Figures 4(c) and 4(d)). In the brown adipose tissue between the shoulders, FSP27, HSL, p-HSL/HSL, CGI-58, and ATGL were higher in SG and RYGB than in sham and control rats 2 and 4 weeks following surgery. DGAT1 and DGAT2 were always lower in the bariatric surgery group (Figures 4(e) and 4(f)). The above results show that following the body weight decrease and food intake recovery after weight loss, the concentration of FSP27 protein in WAT and fat hydrolase content changed from low to high, all of which was higher than in obese controls and sham-operated rats. Triglyceride synthase was only reduced from mild to near-obese (control) rat levels. Upregulated FSP27 in brown fat between the scapulae precedes the appearance of white fat, and the persistently higher expression of lipolytic enzymes suggests that brown fat is constantly in an active hydrolysis state within 4 weeks of bariatric surgery. The rapid weight decline then gradually slowed after surgery, suggesting that FSP27 is highly expressed in adipose tissue for a specific period of time, inhibiting fat hydrolysis by regulating the lipolytic enzymes HSL and ATGL and that it may affect the rate of body weight decline in rats.

### 3.5. FSP27 Was Inhibited in 3T3-L1 Adipocytes in High-Fat, High-Sugar, and High-Nutrient Environments

In the process of weight loss and fat hydrolysis in rats, FSP27 content increased from low to high until the rate of weight loss slowed down. We speculated that FSP27 may protect against the body's lack of nutrients and inhibit excessive fat hydrolysis. To assess the effects of different energy and nutrient factors on FSP27 in adipocytes, we induced 3T3-L1 preadipocytes into mature adipocytes (Figure 5(a)) and cultured them in palmitic acid, high glucose, or high-concentration serum media. Compared with controls, palmitic acid, high glucose, and high-concentration serum environments all reduced FSP27 protein abundance. Interestingly, the high-fat environment showed decreased FSP27 yet no change in HSL or ATGL. In a high glucose environment, decreased FSP27 was accompanied by increased HSL and unchanged ATGL. In a high-nutrient environment, decreased FSP27 was accompanied by increased ATGL and slightly decreased HSL. This shows that the regulation of FSP27 on HSL and ATGL may differ upon different energy and nutrient factors. Immunofluorescence staining (Figure 5(c)) confirmed the differences in FSP27 expression and showed its localization at the surface and cytoplasm of LDs. In summary, these results show that FSP27 is lower in fat cells in high-energy, high-sugar, and high-nutrient environments. Obviously, this change is beneficial to fat decomposition and lipid accumulation. The regulation of lipoylation remains to be further studied. Combined with the results of our animal experiments (Figure 4), we speculate that FSP27 is likely to be an energy-related protein which may affect the storage and decomposition of body lipids.

## 4. Discussion

The short- and long-term effects of bariatric surgery have been defined [27, 28]. In this paper, gastric cuff resection and Roux-en-Y gastric bypass both effectively and rapidly caused reduced fat and weight in rats, with a larger effect seen with Roux-en-Y gastric bypass. The fields of weight loss metabolic surgery have been devoted to the metabolic benefits of the surgery itself for many years [29]. If obese people only undergo calorie restriction, their weight loss is usually lower than expected [30]. Because it is difficult to maintain healthy diet and physical activity habits [31], less than half of those who plan to lose weight reduce body weight more than 10% [30, 32, 33]. Bariatric surgery is currently one of the most effective and long-lasting treatments for moderately and severely obese people [34–36].

Bariatric surgery not only causes a decrease in fat content, but also changes in systemic fat distribution in the human body. Body fat presents important metabolic and cardiovascular risk factors, with the proportion of abdominal fat around the hips related to disease associated with obesity and mortality [37]. It is reported that in contrast to central (abdominal) fat, peripheral (hip) subcutaneous fat deposition is protective for insulin resistance [38], visceral obesity, and impaired blood sugar control at the core of metabolic syndrome, increasing the risk of cardiovascular disease [39–41]. In this study, we found that the fat redistribution in rats during the consumption process may have a protective effect for the body, which is conducive to insulin resistance in rats with a high-fat diet.

FSP27 can promote the aggregation of LDs and play an independent and important role in promoting LD fusion and antifat lipolysis [6–8, 10–16, 42, 43]. In mice, loss of FSP27 reduces fat mass and induces the formation of multichamber LDs in white fat cells [44]. FSP27 expression is positively correlated with insulin sensitivity (HOMA-IR index) in human white fat [45]. Destruction of the CIDE-C domain in FSP27 is closely related to human lipodystrophy syndrome, usually leading to ectopic lipid accumulation, dyslipidemia, and insulin resistance diabetes [44]. Many studies show that calorie intake is related to FSP27 expression [19, 20, 46], and the up/downregulation of FSP27 is an adaptive change of fat cells following an oversupply or insufficiency of systemic energy and nutrients [20, 21]. In this study, food intake of rats after SG and RYGB was lower than that of obese rats, and the expression of FSP27 in white fat was lower than in control rats after operation. At four weeks after bariatric surgery, the expression of FSP27 in white fat was higher than that in obese rats, although the weight and body fat were still lower than that in obese control rats. FSP27 expression in brown adipose tissue was always higher after operation than in obese control rats, showing that weight reduction surgery also affects lipid metabolism by limiting caloric intake. FSP27 is associated with a variety of pathways and behaviors of lipid metabolism: it is involved in fat hydrolysis, white fat “browning” [47], and even fat autophagy by regulating the function of fat hydrolase and changing the morphology of LDs [48]. FSP27 also promotes LDs fusion independent of fat hydrolysis [13]. Therefore, different FSP27 content in the fat of rats with weight loss may influence many factors.

The expression of ATGL, HSL, and DGAT can be indicators for evaluating lipid synthesis and decomposition. ATGL increased in the gonadal white fat (GWAT) of mice with FSP27 knocked out [18], indicating that FSP27 interacts directly with ATGL to inhibit its activation [15]. The acute damage caused by siRNA against FSP27 in differentiated white fat cells led to increased Lipe (HSL) mRNA [8]. These studies show that FSP27 affects fat hydrolysis by inhibiting ATGL and HSL expression. In our study, FSP27 expression in white fat (epididymis and renal circumference fat) in rats after SG and RYGB changed from low to high, and the expression of HSL, p-HSL/HSL, ATGL, and CGI-58 changed from high to low (Figure 4). This supports the inhibitory effect of FSP27 on fat hydrolase in vivo and corresponds to FSP27 changes in body weight from a rapid decline into a relatively stable state (Figure 1(b)). The decrease in FSP27 expression at 2 weeks after weight loss may be related to the limited caloric intake caused by bariatric surgery, and its decrease reduced the inhibition of fat hydrolase, at which point the rat weight decreases continuously and rapidly. The expression of FSP27 in thin rats was pronouncedly higher than in obese control rats at 4 weeks after operation, and this change slowed down fat consumption and tended to restore fat hydrolysis and synthesis to a kind of “balance”. DGAT1 and DGAT2 were reduced from early mild to near normal levels, and this “balance” was achieved to some extent by FSP27 regulation of fat hydrolase rather than synthase. A previous study found that lipid hydrolysis of isopropyl adrenaline paradoxically increased FSP27 protein in 3T3-L1 fat cells, suggesting that the FSP27 increase was used as a feedback mechanism to inhibit excessive lipids induced by powerful beta-adrenaline stimulation [13]. The rapid reduction of adipose tissue following weight reduction surgery alludes to a similar strong lipid solution. We speculate that this feedback increase of FSP27 is a kind of “protective” function which prevents excessive fat hydrolysis and weight reduction after operation. This “protective” effect may explain why patients cannot lose weight to the desired level after bariatric surgery and may even regain weight [28, 49]. The effect of FSP27 on lipid metabolism changes during this period is worthy of further study.

Alternatively, there are reports that FSP27 may locate LD-LD contact sites (LDCS) and mediate the flow of lipids from small LDs to large lipid titration, forming larger LDs [12]. Our immunohistochemistry (Figure 3) showed that thin rats have more LDs and higher FSP27 expression. This study showed that after bariatric surgery there are more little LDs and UCP1 mRNA is upregulated in white and brown fat in thin rats, suggesting the process of “browning” white adipose tissue initiates. The formation of multicellular LDs depends on FSP27 function [47]. Therefore, after bariatric surgery FSP27 expression was increased in white fat cells in the trunk of rats.

It has been reported that the change in FSP27 can combat the excessive hydrolysis and accumulation of adipose tissue, and FSP27 was reduced in the adipose tissue of obese individuals [22, 50]. We found that 3T3-L1 cells in media with high-fat, high-sugar, and high-serum concentration reduced FSP27 expression. Combined with our animal experiments (Figure 4), this suggests that FSP27 is downregulated when nutrients are relatively abundant and FSP27 is upregulated when nutrients are lacking.

In summary, our study reveals that FSP27 plays a role in lipid breakdown and storage in the body, which is regulated by energy and nutrient supply. FSP27 can inhibit fat breakdown by inhibiting HSL and ATGL expression and mediating LDs formation. This study provides a potential treatment for clinical morbid obesity after bariatric surgery.

## Figures and Tables

**Figure 1:** Changes in food intake, body weight, and TG content in plasma and adipose tissue in different groups of rats. Rats were given a high-fat diet and water* ad libitum*. Average daily feeding weight (a) was recorded. Body weight (b) was measured at 0, 7, 14, 21, and 28 days after surgery in each group. TG levels were measured in plasma (c) and adipose tissue (d). Control: obese rats, sham: obese and sham-operated, SG: obese rats undergoing gastric sleeve resection, and RYGB: obese rats receiving Roux-En-Y gastric bypass. Data are expressed as $\overset{-}{x}$  ± SD: 8 rats in SG group and 10 rats in each remaining group. *∗*=P <0.05 versus control group, #=P <0.05 versus sham group.

**Figure 2:** The body composition of rats was determined by dual-energy X-ray absorptiometry. Fat mass (b) and lean mass (c) were analyzed separately. Further examination of body fat/body weight (%) (d), (upper limb + thigh)/trunk fat (e), and trunk/body fat ratio (%) (f). Data are expressed as $\overset{-}{x}$  ± SD; *∗*=P <0.05 versus control group; #=P <0.05 versus sham group.

**Figure 3:** Trunk fat in postoperative rats was detected by immunohistochemical staining and real-time RT-PCR. Immunohistochemical staining of FSP27, original magnification × 400 (a). Relative expression levels of Fsp27 (b) and UCP1 (c) mRNA in brown fat between epididymis, perirenal, and scapular. Data are expressed as $\overset{-}{x}$  ± SD; *∗*=P <0.05 versus control group; #=P <0.05 versus sham group.

**Figure 4:** Protein expression in trunk fat at 2 and 4 weeks after surgery detected by western blotting. Representative images of FSP27, HSL, P-HSL/HSL, ATGL, CGI-58, DGAT1, DGAT2, and *β*-catenin in epididymal fat at 2 and 4 weeks, and grayscale contrast internal reference (a). Perirenal fat representative expression of each protein and grayscale contrast internal reference value (b). Representative expression of each protein in the interscapular fat and grayscale contrast internal reference value (c). Data were expressed as $\overset{-}{x}$  ± SD; *∗*=P <0.05 versus control group; #=P <0.05 versus sham group.

**Figure 5:** The expression and localization of FSP27 in 3T3-L1 cells in different energy and nutrient environments. 3T3-L1 cell were induced to maturity by medium I (containing 10 ml FBS, 89 ml DMEM/F12 liquid medium, 1 ml streptomycin, 1 mg/L bovine insulin, 0.5 mmol/L IBMX, and 1.0 *μ*mol/ L DEX) and induced to differentiation by medium II (containing 10 ml FBS, 89 ml DMEM/F12 liquid medium, 1 ml streptomycin, and 1 mg/L bovine insulin). Cells were visualized with Oil Red O staining (a). Cells were then cultured with high-fat, high-sugar, high-serum, or control medium separately for 48 hours, and FSP27 was detected by western blotting (b) and immunofluorescence (c). *∗* indicates P<0.05;* ns* indicates P>0.05.

**Table 1:** Gene-specific primers for real-time RT-PCR analysis.

Gene		Primer sequence
FSP27	Forward	GCCCGGGTAACCTTTGACCT
	Reverse	GCGGAGCATTTCCTTCACGA
UCP1	Forward	ACTGCCACACCTCCAGTCATT
	Reverse	CTTTGCCTCACTCAGGATTGG
*β*-actin	Forward	GGAGATTACTGCCCTGGCTCCTA
	Reverse	GACTCATCGTACTCCTGCTTGCTG

## Data Availability

The data used to support the findings of this study are available from the corresponding author upon request.
